RETRACTED

# Feature Extraction of Ancient Chinese Characters Based on Deep Convolution Neural Network and Big Data Analysis

**DOI:** 10.1155/2021/2491116

**Published:** 2021-08-30

**Authors:** Cheng Zhang, Xingjun Liu

**Affiliations:** ^1^College of Literature and Journalism, Chengdu University, Chengdu 610106, Sichuan, China; ^2^School of Humanities and Communication, Sanya University, Sanya 572022, Hainan, China

## Abstract

In recent years, deep learning has made good progress and has been applied to face recognition, video monitoring, image processing, and other fields. In this big data background, deep convolution neural network has also received more and more attention. In order to extract the ancient Chinese characters effectively, the paper will discuss the structure model, pool process, and network training of deep convolution neural network and compare the algorithm with the traditional machine learning algorithm. The results show that the accuracy and recall rate of the Chinese characters in the plaque of Ming Dynasty can reach the peak, 81.38% and 81.31%, respectively. When the number of training samples increases to 50, the recognition rate of MFA is 99.72%, which is much higher than other algorithms. This shows that the algorithm based on deep convolution neural network and big data analysis has excellent performance and can effectively identify the Chinese characters under different dynasties, different sample sizes, and different interference factors, which can provide a powerful reference for the extraction of ancient Chinese characters.

## 1. Introduction

As one of the oldest languages in the world, ancient Chinese characters have a long cultural history and have a great influence on the production of other languages. In the deep analysis of ancient Chinese characters, the first step is to extract the relevant features. In order to extract the features of ancient Chinese characters effectively, we need to use the corresponding algorithm as a research means. Li et al. proposed a data prediction method based on deep convolution neural network to solve the problem that it is difficult to obtain accurate physical model for system prediction in most cases and carried out corresponding prediction experiments. The results show that this method can effectively ensure the accuracy of prediction [1]. Mokhtia et al., aiming at the problem of feature selection, ridge method, cable method, and elastic network regression method, used to explore it, and fuzzy correlation matrix is added to its objective function. Finally, the minimum redundancy of features is successfully solved, and the effectiveness of fuzzy correlation matrix is verified [2]. Alfarraj found that the core purpose of the intelligent transportation system is to maintain road safety, in which road crack detection is extremely important. By proposing an IOT system based on the deep learning method of biological stimulation, the pixel accuracy, prediction accuracy, and recall rate of road crack detection are guaranteed [3]. Najafzadeh et al. applied the artificial intelligence model to explore the scouring depth under the action of stable current and realized the effective prediction of scouring depth and scouring trend under different conditions by constructing the nonlinear regression equation of maximum equilibrium scouring depth [4].

RETRACTED

Wei et al. proposed an improved convolution neural network algorithm based on depth, aiming at the problems of small target loss, rough edge, and poor semantic segmentation in the traditional algorithm of extracting buildings from high-resolution remote-sensing images, and realized pixel level end-to-end semantic segmentation through model fusion strategy [5]. Gan et al. found that neural network provides a new method for facial beauty prediction, but there are some problems such as less public databases and high subjectivity of facial appearance evaluation. Therefore, a feature extraction model based on illumination depth convolution neural network is constructed, which significantly improves the classification accuracy of facial beauty prediction [6]. Yang et al. believe that crack detection is the key to ensure the safety of bridges, highways, and other infrastructure. Accordingly, a transfer learning method based on deep convolution neural network is proposed, which successfully realizes the effective detection of cracks. This method has high detection accuracy and comprehensiveness [7]. A new method for detecting the new crown pneumonia by using deep convolution neural network was developed. By integrating deep learning and performance indicators (accuracy, recall, specificity, accuracy, and F1 fraction), the overall accuracy and sensitivity were ensured [8].

Ren et al. proposed a malware visualization method based on deep convolution neural network for the problem of malware visualization. The visualization was verified by space filling curve mapping, Markov point graph, and other methods. The method showed a high malware detection accuracy [9]. Nguyenet et al. applied deep convolution neural network to document digital segmentation, using rough classifier and fine combination classifier to recognize each character pattern, and achieved significant recognition and segmentation effect [10]. Shen et al. aimed at the problems of high computational complexity and large amount of computation of deep convolution neural network, combined the feature representation learnt from the object-oriented dataset and the scene-centered dataset, constructed a new target detection framework, and successfully improved the detection accuracy [11]. Jin et al. used the deep convolution neural network to realize the denoising of the chest X-ray image. Through the residual learning of noise distribution, the convergence speed of the network model was effectively accelerated, and a good denoising effect was achieved [12].

RETRACTED

To sum up, the deep convolution neural network is widely used in various fields and has achieved good model prediction effect, with high prediction accuracy. In the context of big data, deep convolution neural network can be further optimized. In view of this, this experiment will explore the feature extraction of ancient Chinese characters based on deep convolution neural network and big data analysis, in order to improve the feature recognition and extraction ability of the model.

## 2. Feature Extraction Algorithm Based on Deep Convolution Neural Network

### 2.1. Model Structure and Pooling Process of Deep Convolution Neural Network

Aiming at the problem of feature extraction of ancient Chinese characters, this subject experiment deeply explores it in combination with deep convolution neural network and big data analysis. The research process of this subject experiment is shown in Figure 1.

According to Figure 1, this subject experiment will focus on the analysis of deep convolution neural network, explore its network model structure, pooling process, and network training in turn, and apply it to the extraction of ancient Chinese characters, so as to realize the quantitative analysis of its detection and extraction performance. When extracting the features of Chinese characters from different dynasties in the experiment, various image acquisition tools including sensors need to be used.  Figure 2 shows the sensors applied in the experiment.

In deep neural network (DNN), convolution neural network (CNN) with local receptive field and downsampling structure is the most widely used one [13]. Compared with other DNNS, CNN can significantly improve the speed of network training, reduce the network structure parameters, and reduce the use of computing resources. The deep convolution neural network (DCNN) can be obtained by organically combining the two network models to further optimize the performance of feature recognition and extraction [14]. DCNN includes the convolution layer and the pooling layer, and each network layer is alternately superposed. Its network model is shown in Figure 3.

In Figure 3, *Ci* represents the convolution layer, *Si* represents the lower sampling layer, and *i* is the network layer serial number. Therefore, there are three convolution layers in the DCNN network model, namely, *C*1, *C*3, and *C*5, two pooling layers, *S*2 and *S*4, respectively, and a fully connected layer *F*6 [15]. The black-and-white plane represents the feature map extracted by the network model, and there are some differences among the feature maps. In any convolution layer, the convolution kernel will generate sliding convolution with the output result of the previous layer and then generate all the feature pixel values contained in the feature map. The calculation formula is shown as follows:

(1) $$\begin{array}{c} y_{pj}^{\left(l\right)}=f\left(\sum_{i\in M_{j}^{\left(l-1\right)}}\sum_{\left(u,v\right)\in K^{\left(l\right)}}W_{ij\left(u,v\right)}^{\left(l\right)}\circ X_{pi}^{\left(l-1\right)}\left(c+u,r+v\right)+b_{j}^{\left(l\right)}\right), \end{array}$$

where *W*_*ij*_^(*l*)^ is the convolution kernel, *b*_*j*_^(*l*)^ is the offset of the *j* characteristic graph of the *l* layer, *c* and *r* and *u* and *v* are variables, and the former represents the vertical and horizontal feature pixels, respectively, while the latter represents the vertical and horizontal step size of *W*_*ij*_^(*l*)^, respectively, *K*={(*u*, *v*) ∈ *N*^2^*|*0 ≤ *u* ≤ *k*_*x*_; 0 ≤ *v* ≤ *k*_*y*_}, *k*_*x*_ and *k*_*y*_ represent the length and width of *W*_*ij*_^(*l*)^ in the *l* layer, respectively, *f* is the activation function of the *l* layer, and *p* is the *p* training sample. In the pooling layer, the pooling window performs sliding sampling in the feature graph output from the previous layer, thus generating all the feature pixel values of the feature graph in the network layer:

(2) $$\begin{array}{c} y_{pj}^{\left(l\right)}=\left(\frac{\sum_{\left(u,v\right)\in S^{l}}x_{pi}^{\left(l-1\right)}\left(c+u,r+v\right)}{\left(s_{x}\cdot s_{y}\right)}\right), \end{array}$$

where *S*^(*l*)^={(*i*, *j*) ∈ *N*^2^*|*0 ≤ *u* ≤ *s*_*x*_^(*l*)^, 0 ≤ *v* ≤ *s*_*y*_^(*l*)^} and *s*_*x*_^(*l*)^ and *s*_*y*_^(*l*)^ represent the length and width of the downsampling window in layer *l*, respectively. Common pooling operations are divided into average pooling operation and maximum pooling operation. The former is to add all the characteristic pixel values in the pooling window and then divide them by the number of pixels to obtain the average value in the pooling layer. The latter refers to comparing and analyzing all the characteristic pixel values in the pooling window, sampling the maximum value, and finally taking it as the characteristic pixel value of the maximum pooling processing [16]. Two different pooling processes are shown in Figure 4.

RETRACTED

Figure 4(a) shows the average pooling operation. The four colors in the upper generous box represent four different pool areas, respectively, and the lower colors represent the corresponding sampling values after the average pooling treatment. Taking the blue area of Figure 4(a) as an example, the four characteristic pixels of pool region are 3, 4, 4, and 5, respectively, and the number of pixels is 4; then, the sample value below can be obtained as 4. Figure 4(b) is the maximum pool operation, similar to Figure 4(a). The four colors of the upper big box represent different pool areas, respectively. After the maximum pool processing, the sampling value corresponding to the small box below can be obtained. Taking green area as an example, before the maximum pool processing, the four characteristic pixels in the region are 7, 8, 3, and 8, respectively. If the maximum window value is selected, the sampling pixel value after the maximum pooling processing is 8. The eigenvalue value of the maximum pool operation can be calculated by the following formula:

(3) $$\begin{array}{c} \max\left(x_{pi}^{\left(l-1\right)}\left(c+u,r+v\right)\right). \end{array}$$

### 2.2. Training of Deep Convolution Neural Network Based on Loss

Deep convolution neural network can be divided into two types, namely, neural network with loss function and neural network without loss function. The former has more extensive applicability [17–19]. For the deep convolution neural network with loss function, the core idea is to train the convolution kernel by gradient descent [10, 20–22]. The main methods include automatic coder training, restricted Boltzmann machine training, and overall model training based on reverse feedback. Due to the limited space, this experiment only focuses on the training methods of the automatic coder. This method is an effective convolution kernel training method, which can deeply learn the abstract features without supervision. Its basic structure is shown in Figure 5.

According to Figure 5, the basic structure of the automatic coder includes three parts: input layer, hidden layer, and output layer. Through the input layer, the relevant data is transmitted to the hidden layer, which is the coding process. The stage of data transmission from the hidden layer to the output layer is called the decoding process. Let the training vector be $\overset{⟶}{x}$ and $\overset{⟶}{x}=\left\{x_{1},x_{2},x_{3},\ldots \right\}$. The hidden layer is expressed as $\overset{⟶}{h}$. The output layer is represented as $\tilde{x}$. The mapping formula of coding process is shown in the following equation:

(4) $$\begin{array}{c} \overset{⟶}{h}\left(\overset{⟶}{x}\right)=f\left(W\overset{⟶}{x}+\overset{⟶}{b_{h}}\right), \end{array}$$

where *f* is the activation function, *W* is the weight matrix in the encoding process, and $\overset{⟶}{b_{h}}$ is the offset vector in the input layer. After encoding, the input original data is mapped into the corresponding feature vector, which can be decoded. The mapping formula is shown in the following equation:

(5) $$\begin{array}{c} \overset{⟶}{x}=f\left(W^{T}\overset{⟶}{h}\left(\overset{⟶}{x}\right)+\overset{⟶}{b_{r}}\right), \end{array}$$

where *W*^*T*^ represents the weight matrix in the decoding process and its value is consistent with the transpose of *W* and $\overset{⟶}{b_{r}}$ is the offset vector contained in the hidden layer. Since the automatic encoder is an unsupervised learning neural network training model, the purpose of its network training is to make the target value consistent with the initial input value; then, the overall loss function, as shown in equation (6), can be obtained:

(6) $$\begin{array}{c} J_{\text{AE}}\left(\theta \right)=\sum_{\overset{⟶}{x}\in D}L\left(\overset{⟶}{x},\overset{⟶}{r}\right), \end{array}$$

where *J*_AE_(*θ*) is the loss function, *D* is the set of all training vectors, and *L* is the error in training. As the main function of the loss function is to show the approximate degree of input and output, in order to get the maximum value, we usually need to use the gradient descent method *J*_AE_(*θ*) to optimize; see equation (7), for details:

(7) $$\begin{array}{c} \theta =\theta -\lambda \nabla \theta . \end{array}$$

Equation (7) can update the relevant parameters, where *λ* is the step size and ∇*θ* is the gradient value of the parameters. Because there is a difference between the probability of the model classifier and its corresponding label, there will be a gradient in the network training, according to which the output layer error formula, as shown in equation (8), can be obtained:

(8) $$\begin{array}{c} \delta^{o}=f^{\prime }{\left(W^{T}\overset{⟶}{h}\left(\overset{⟶}{x}\right)+\overset{⟶}{b_{r}}\right)}^{T}\left(\overset{⟶}{x}-x\right), \end{array}$$

where *δ*^*o*^ represents the error in the output layer of the network, from which the error in the hidden layer can be obtained:

(9) $$\begin{array}{c} \delta^{h}=\left(W\delta^{o}\right)f^{\prime }\left(W\overset{⟶}{x}+\overset{⟶}{b_{h}}\right). \end{array}$$

Similarly, *δ*^*h*^ represents the error in the hidden layer; then, the weight matrix *W* can be calculated by

(10) $$\begin{array}{c} \nabla W=f\left(W\overset{⟶}{x}+\overset{⟶}{b_{h}}\right)\delta^{h}. \end{array}$$

RETRACTED

## 3. Feature Detection and Extraction of Chinese Characters Based on Deep Convolution Neural Network

### 3.1. Target Detection Parameters and Evaluation Indexes

In the detection of Chinese character target features, measurement parameters need to be used to accurately evaluate the detection performance [23–25]. IoU, as a parameter that can give the closeness of the prediction object between the prediction region and the real region, plays an important role in it. First, you need to define four values, as shown in Table 1.

According to Table 1, IoU can be defined, and its calculation formula is shown as follows:

(11) $$\begin{array}{c} \text{IoU}=\frac{\text{TP}}{\text{FP}+\text{TP}+\text{FN}}. \end{array}$$

It can be seen from equation (11) that the IoU score is a measure based on counting, and the output of deep convolution neural network is a probability value, which can be used to indicate that the region is essentially a part of the detection object. Therefore, there is a deviation in the calculation of the IoU score by using the output of neural network, and the probability value is usually used to approximate the IoU score. Then, the precision rate and recall rate can be defined, and the former is shown as follows:

(12) $$\begin{array}{c} \text{Precision}=\frac{\text{TP}}{\text{TP}+\text{FP}}. \end{array}$$

The accuracy rate Precision is the ratio of TP to all the targets judged as positive samples, and the formula of recall rate is shown as follows:

(13) $$\begin{array}{c} \text{Recall}=\frac{\text{TP}}{\text{TP}+\text{FN}}. \end{array}$$

The recall rate Recall in equation (13) represents the ratio of TP to all positive samples with true values. If the Chinese character data samples to be predicted are all negative samples, then according to formulas (12) and (13), Precision and Recall are both 0. Therefore, in this case, only relying on Precision and Recall cannot achieve the evaluation of the effectiveness of Chinese character target detection. It is very necessary to maintain the balance between the two. Different Precision and Recall can be generated by setting a differentiated threshold, and the PR curve can be obtained. See Figure 6, for details.

For any target detection algorithm model, when its Precision and Recall are higher, its detection accuracy can also reach a higher value. However, Precision and Recall usually show the opposite state. If Precision is high, Recall is relatively low, and vice versa. The area surrounded by the PR curve can represent the performance of the prediction model [26–28]. When the target to be detected is located, the method of border regression is usually used. The size and position of the target can be effectively adjusted by modifying the border of the candidate region, as shown in Figure 7.

RETRACTED

In Figure 7, *P* represents the target border output by the target detection algorithm model, *G* represents the real Border marked and determined, and the regression of the border can be realized by functional transformation so that the border $\hat{G}$ and *G* after regression processing are closer. First of all, a window needs to be translated so that the center coordinate of the window changes from (*x*, *y*) to (△*x*, △*y*), and △*x*=*P*_*ω*_*d*_*x*_(*P*) and △*y*=*P*_*h*_*d*_*y*_(*P*) have the formula

(14) $$\begin{array}{c} {\hat{G}}_{x}=P_{\omega }d_{x}\left(P\right)+P_{x},\\ {\hat{G}}_{y}=P_{h}d_{y}\left(P\right)+P_{y}, \end{array}$$

where *ω* and *h* represent the width and height of the window, respectively. Then, scaling is performed:

(15) $$\begin{array}{c} {\hat{G}}_{\omega }=P_{\omega }\exp\left(d_{\omega }\left(P\right)\right),\\ {\hat{G}}_{h}=P_{h}\exp\left(d_{h}\left(P\right)\right). \end{array}$$

In essence, the input box *P* of border regression is a convolution feature vector corresponding to the border. After translation and scaling, *P* generates a transformation, and the predicted value $\hat{G}$ of Chinese characters can be obtained.

### 3.2. Feature Detection and Extraction of Chinese Characters

Common target detection algorithms are usually difficult to achieve efficient feature expression, while deep learning can meet the needs of target detection in many cases [29–31]. Two-step detection algorithm is often used to detect targets. Based on generating candidate regions, detection results are obtained by regression processing. The algorithm structure is shown in Figure 8.

Figure 8 shows that, on the basis of CNN, a ROI pooling layer is added to the two-step detection algorithm based on deep learning, which can apply the multitask loss function to complete the effective classification and location. It not only retains more feature information as much as possible but also simplifies the amount of computation. The algorithm is divided into three steps: feature extraction, candidate region generation, and target location. The process of feature extraction is consistent with that of traditional CNN, which will not be described here. Candidate region generation refers to the preliminary generation of some candidate regions and distinguishes them and judges that the region is the foreground or background if it is the foreground, then reserve it. On the contrary, it is ignored. In the Chinese character target feature map, nine panes will be generated in any pixel, and each pane has different scales. Therefore, any feature map contains 9 × *H* × *W* panes; *H* and *W* represent the depth and width of the feature map, respectively. After all the panes have been marked, the approximate position of the foreground of Chinese character target feature can be obtained by border regression processing, which indicates that the preliminary candidate region has been generated. In the network training of two-step detection algorithm based on deep learning, and its classification module and border regression module need to be jointly processed; that is, the loss function of the two modules should be jointly trained, and the loss function in the training network can be expressed as

(16) $$\begin{array}{c} L\left(\left\{p_{i}\right\},\left\{u_{i}\right\}\right)=\frac{1}{N_{\text{cls}}}\sum_{i}L_{\text{cls}}\left(p_{i},p_{i}^{*}\right)+\lambda \frac{1}{N_{\text{reg}}}\sum_{i}p_{i}^{*}L_{\text{reg}}\left(t_{i},t_{i}^{*}\right), \end{array}$$

where*N*_cls_ represents the size of a transmission channel, and its value is 256, *L*_cls_(*p*_*i*_, *p*_*i*_^*∗*^) is the logarithm loss value of the target foreground and background, *p*_*i*_ is the probability that the pane is predicted as the target, and *p*_*i*_^*∗*^ is 1. The average of all the loss values in a transmission channel can be calculated to obtain the loss of the training network. *N*_*reg*_ is the total number of panes contained in it, *λ* is the balance ratio of the two losses, *t*_*i*_ is the output result of the border regression module, and *t*_*i*_^*∗*^ is the offset between any pane and the real value during the network training.

RETRACTED

## 4. Experimental Results and Analysis

### 4.1. Feature Extraction of Ancient Chinese Characters Based on Deep Convolution Neural Network

In this experiment, four ancient Chinese characters of Tang Dynasty, Song Dynasty, Yuan Dynasty, and Ming Dynasty are selected to carry out the feature extraction experiment. The Chinese character information of each dynasty is taken as the input content, including four different positions of Chinese characters in paper, bamboo slips, stone tablets, and plaques. Four corresponding vectors are generated to carry out network training and feature extraction. The results are shown in Figure 9.

Figure 9 shows that the performance of ancient Chinese character feature extraction based on deep convolution neural network is different in recognizing and extracting characters of different dynasties. According to Figure 9, the accuracy and recall rate of the method proposed in this experiment are high, which can be maintained at about 80%, and the accuracy and recall rate can reach the highest value, 81.38% and 81.31%, respectively, when recognizing the characters in the plaque. Secondly, the recognition accuracy of Yuan Dynasty Chinese characters is higher than 75%, and the highest value is 79.54% when recognizing the characters on the plaque. When recognizing Chinese characters on bamboo slips, the recall rate can reach 78.44%. The average accuracy rate and recall rate of Chinese character recognition in Tang Dynasty rank third, about 70%. The accuracy and recall rate of the algorithm proposed in this experiment are lower than 70%, and the lowest value is 67.78%. The lowest value of the latter is 70.33%. In the comparison of the speed and accuracy of network model training, this experiment will take the recognition of ancient Chinese characters on the plaque as an example, and the changes of the results are shown in Figure 10.

RETRACTED

As can be seen from Figure 10, with the progress of network training, the accuracy rate, recall rate, the harmonic average of accuracy rate, and the recall rate of the model show a trend of first increasing and then flattening. When the number of training is less than 10 times, the three show an exponential growth trend. Then, the growth rate is gradually decreased. When the network model is trained about 40 times, the accuracy of the model is almost stable, and the convergence speed of the model is fast. This shows that the feature extraction algorithm of ancient Chinese characters based on deep convolution neural network has superior performance and can realize the effective recognition and extraction of ancient Chinese characters.

### 4.2. Comparison of Feature Extraction Rate between Deep Convolution Neural Network and Other Algorithms

In order to objectively evaluate the performance of ancient Chinese character feature extraction algorithm based on deep convolution neural network, this experiment applies this algorithm and other algorithms to train samples with different sample sizes. The algorithms involved in the experiment include three traditional machine learning algorithms, namely, MFA, PCA, and LDA. The recognition rate of Chinese character feature is shown in Figure 11.

Figure 11 clearly shows that compared with the traditional machine learning algorithm, the deep convolution neural network algorithm based on deep learning has higher recognition rate of Chinese characters. With the increasing number of training samples, the recognition rates of the four algorithms are improving. When the number of training samples is 5, the recognition rate of DCNN is 81.35%, which is significantly higher than that of MFA, PCA, and LDA. The recognition rates of these three algorithms are 66.06%, 60.61%, and 67.31%, respectively. When the number of training samples reaches 50, the recognition rate of MFA, PCA, and LDA is 97.21%, 94.32%, and 97.49%, respectively, while the recognition rate of deep convolution neural network algorithm is as high as 99.72%. In the case of adding certain occlusion or noise interference, the comparison results of the four algorithms are shown in Figure 12.

RETRACTED

As can be seen from Figure 12, with the continuous growth of occlusion rate, the recognition effect of all algorithms shows varying degrees of decline. The descending trend of PCA algorithm is very significant. The descending rate of MFA algorithm and LDA algorithm is slightly lower than that of PCA algorithm, but still significantly higher than that of deep convolution neural network algorithm. When the occlusion rate increases to 70%, the recognition rate of deep convolution neural network algorithm can still reach more than 50%, and its value is 58.87%. Under the condition of salt and pepper and Gaussian noise, the recognition rate of the proposed algorithm is 10.32% and 8.74%, respectively, which is much higher than MFA, PCA, and LDA. This shows that although the continuous improvement of occlusion rate and noise will reduce the recognition rate of the algorithm proposed in this experiment, compared with other traditional machine algorithms, the ancient Chinese character feature recognition algorithm based on deep convolution neural network still has better extraction performance, showing higher recognition rate and accuracy.

## 5. Conclusion

With the continuous development of deep learning, more and more feature extraction algorithms take deep learning as the core technology. With its unique structural advantages, deep convolutional neural network has become one of the most widely used feature extraction methods. In order to extract the features of ancient Chinese characters accurately, this experiment takes the deep convolution neural network algorithm as the research focus, deeply explores its model structure, pooling process, and network training, and applies it to the extraction of ancient Chinese characters. In addition, the deep convolution neural network algorithm is compared with other algorithms to explore the effect of feature recognition and extraction of various algorithms under different influencing factors. The results show that the recognition rate of this algorithm is higher than other algorithms in the recognition of Chinese characters in Tang, Song, Yuan, and Ming Dynasties, and the highest accuracy and recall rate can reach 81.38% and 81.31%, respectively. The recognition rate of ancient Chinese character feature extraction algorithm based on deep convolution neural network can be improved with the increase of sample size, and the increase is significantly greater than other traditional machine learning algorithms. When the training sample size is 50, the recognition rate is as high as 99.72%. When the interference factors are increasing, the feature extraction algorithm of ancient Chinese characters based on deep convolution neural network can still maintain a high recognition rate. The method proposed in this subject experiment can provide strong technical support for the feature extraction of ancient Chinese characters, promote the society to further explore the ancient civilization, and also provide a certain reference for the feature extraction in other fields. The novelty of this research is that the deep convolution neural network is applied to the feature extraction of ancient Chinese characters for the first time, which provides a certain reference for the recognition and extraction of ancient Chinese characters. Compared with the traditional feature extraction methods, the algorithm is more novel and efficient. Although we have obtained some research results in this experiment, when we analyze the training model of deep convolution neural network, we do not analyze the situation of no loss function in detail. We hope to improve it in the future. The training model of deep convolution neural network without loss function is further explored.

RETRACTED

## Figures and Tables

**Figure 1:** Research flow of ancient Chinese character feature extraction based on deep convolution neural network and big data analysis.

**Figure 2:** Sensor used for image acquisition.

**Figure 3:** Schematic diagram of the DCNN network model.

**Figure 4:** Common pooling process diagram. (a) Average pooling operation and (b) maximium pooling operation.

**Figure 5:** Structure diagram of the automatic encoder.

**Figure 6:** Schematic diagram of the PR curve.

**Figure 7:** Schematic diagram of border regression.

**Figure 8:** Structure of two-step detection algorithm based on deep learning.

**Figure 9:** Ancient Chinese character feature extraction results.

**Figure 10:** The change rate of the experimental results of recognizing the characteristics of ancient Chinese characters on plaques.

**Figure 11:** Comparison of recognition rate of Chinese characters between deep convolution neural network and traditional machine learning algorithm under different training samples.

**Figure 12:** Comparison of recognition rate of Chinese characters between deep convolution neural network and traditional machine learning algorithm under different occlusion and interference.

**Table 1:** Numerical definition in Chinese character target detection.

The real situation		A case in point	Counterexample
Forecast results	A case in point	TP (real positive example)	FP (false positive example)
	Counterexample	FN (false counterexample)	TN (true counterexample)

RETRACTED

## Data Availability

The data used to support the findings of this study are available from the corresponding author upon request.
